This article has been retracted.

# Effects of Dapagliflozin in Combination with Metoprolol Sustained-Release Tablets on Prognosis and Cardiac Function in Patients with Acute Myocardial Infarction after PCI

**DOI:** 10.1155/2022/5734876

**Published:** 2022-08-03

**Authors:** Hao Zhang, Zeyan Liu

**Affiliations:** Department of Emergency Medicine, The Second Affiliated Hospital of Anhui Medical University, Hefei, Anhui 230601, China

## Abstract

**Objective:**

To find the effects of dapagliflozin in combination with metoprolol sustained-release tablets on cardiac function and prognosis in acute myocardial infarction patients after PCI.

**Methods:**

A total of 84 patients with myocardial infarction who experienced PCI from February 2020 to February 2022 were included and allocated into 3 groups: groups A, B, and C (*n* = 28/per group). Group A was given dapagliflozin combined with metoprolol sustained-release tablets, group B was given dapagliflozin, and group C was given the placebo. Left ventricular end diastolic diameter (EDD), left ventricular ejection fraction (LVEF), and end systolic diameter (ESD) were measured before and after treatment in all groups; myocardial infarction areas were matched among all three groups at 3 months posttreatment. The serum concentrations of interleukin-6 (IL-6), hypersensitive C-reactive protein (hs-CRP), superoxide dismutase (SOD), and malondialdehyde (MDA) were detected in all three groups before and after treatment. The levels of N-terminal probrain natriuretic peptide (NT-pro BNP), lipoprotein (a) (Lp(a)), ischemia-modified albumin (IMA), and secreted frizzled-related protein 5 (SFRP5) were also detected in the serum of all groups. Adverse reactions and cardiovascular adverse events were matched between all groups.

**Results:**

The levels of LVEF in groups A and B were increased after treatment, while the levels of EDD and ESD were decreased. The improvement degree of LVEF and EDD levels in groups A and B was found greater compared to group C (*P* < 0.05). No significant difference was found in myocardial infarction area among the three groups at 3 months postoperation (*P* > 0.05). Serum concentrations of MDA, hs-CRP, IL-6, IMA, NT-proBNP, and Lp(a) were found to decrease in all three groups after treatment, while the levels of SOD and SFRP5 were increased. The improvement degree of serum hs-CRP, IL-6, SOD, MDA, IMA, NT-proBNP, Lp(a), and SFRP5 levels was greater in both groups A and B compared to group C. The improvement degree of serum hS-CRP, SOD, MDA, IMA, Nt-probNP, Lp(a), and SFRP5 levels was significantly greater in group A compared to group B (*P* < 0.05). No adverse effect was observed in all three groups (*P* > 0.05). Total occurrence of cardiovascular adverse effects such as stent thrombosis, heart failure, ventricular fibrillation, and death was 10.71% in group A, 25.00% in group B, and 53.75% in group C. There was statistical significance in the onset of cardiovascular adverse effects 3 months postoperation among all three groups (*P* < 0.05).

**Conclusion:**

Dapagliflozin with metoprolol sustained-release tablets can be effective in improving the heart function, inflammatory response, oxidative stress response, and prognosis in patients after PCI.

## 1. Introduction

Persistent myocardial ischemia and hypoxia caused by coronary artery occlusion can lead to acute myocardial infarction. According to relevant studies, the number of new acute myocardial infarction cases in China can reach 500,000 every year, and the onset age tends to be younger. Percutaneous coronary intervention (PCI) is often used in clinical treatment of acute myocardial infarction, which can quickly open blocked vessels and restore myocardial blood supply. According to the registration data of coronary intervention in mainland China in 2020, there were 968,651 patients undergoing coronary intervention in my country in 2020, ranking first in the world [1]. However, some patients treated with PCI still have poor cardiac function recovery, so it is very important to improve the prognosis of patients with acute myocardial infarction treated with PCI [2–4]. Metoprolol sustained-release tablet is a selective *β*-receptor blocker. According to relevant studies, *β*-blockers can effectively block myocardial inflammation caused by adrenergic receptor activation and can effectively reduce ventricular rate and myocardial oxygen consumption in patients with ischemic cardiomyopathy. They are often used in combination with angiotensin-converting enzyme inhibitors/angiotensin receptor antagonists and other conventional drugs [5, 6]. Dapagliflozin was initially widely used as a hypoglycemic drug in clinic. The mechanism of action of dapagliflozin is that sodium-glucose cotransporter 2 (SGLT2) is expressed in the proximal renal tubules, for the major transporter responsible for glucose reabsorption in renal tubular filtration [7]. According to relevant studies, in addition to its hypoglycemic effect, dapagliflozin can lower blood pressure, diuretic, inhibit myocardial fibrosis, and improve myocardial metabolism and homeostasis [8, 9]. In this study, dapagliflozin combined with metoprolol sustained-release tablets was used in patients with acute infarction undergoing PCI, in order to explore its clinical efficacy.

## 2. Materials and Methods

### 2.1. General Information

A total of 84 patients with myocardial infarction who had undergone PCI from February 2020 to February 2022 were included and randomly separated into three groups: A, B, and C, with 28 patients per group. Four females and 24 males of age from 23 to 87 years were included in group A; the average age was 56.32 ± 12.19 years; 11 cases had diabetes mellitus; 10 cases had heart failure; 11 cases had ventricular arrhythmia; 14 cases had angina pectoris; 12 cases had smoking history. In group B, there were 20 males and 8 females, age from 23 to 86 years old, with an average of 57.68 ± 11.49 years old; 8 cases had diabetes mellitus; 12 cases had heart failure; 15 cases had ventricular arrhythmia; 9 cases had angina pectoris; 16 cases had smoking history. Two females and 26 males of age from 24 to 80 years were included in group C, and the average age was 56.25 ± 12.04 years; 13 cases had diabetes mellitus; 9 cases had heart failure; 10 cases had ventricular arrhythmia; 12 cases had angina pectoris; 15 cases had a smoking history. The three groups' overall data were compared (*P* > 0.05). The present study has been approved by the Hospital Ethics Board.

### 2.2. Inclusion Criteria

① All met the Chinese Medical Association's diagnostic criteria for acute myocardial infarction and were confirmed through imaging. ② The New York Heart Association (NYHA) Classification was grades II to IV. ③ The PCI was carried out within 24 hours of its occurrence. ④ Estimated survival time ≥ 1 year. ⑤ The clinical and imaging data were complete. ⑥ All of them volunteered to participate.

### 2.3. Exclusion Criteria

These are as follows: ① patients allergic to drugs used in this study, ② people with a history of myocardial infarction, ③ patients with severe renal and liver dysfunction, ④ patients with a history of PCI treatment, ⑤ patients with mechanical complications after acute myocardial infarction, ⑥ patients with contraindications to the study drug, and ⑦ patients lost to follow-up.

### 2.4. Methods

Immediately after admission, the patients received general treatment, including ECG, blood pressure, and oxygen saturation detection, bed rest, establishment of venous channels, oxygen inhalation, and correction of water, electrolyte balance, and acid-base balance disorders. Meanwhile, atorvastatin or rosuvastatin was used for plaque stabilization in all three groups. All patients were given oral 300 mg of aspirin (Bayer Health Care Co., Ltd., National drug approval number: J20080078) and 180 mg of ticagrelor (AstraZeneca AB, National drug approval number: J20130020) and then underwent emergency PCI. After PCI, aspirin (100 mg/d) and ticagrelor (180 mg/d) were routinely taken orally. Group C was given placebo, and group B was given dapagliflozin (AstraZeneca Pharmaceuticals Co., Ltd., National drug approval number: J20170040), 10 mg/time, once a day. Group A was given dapagliflozin combined with metoprolol succinate sustained-release tablets (AstraZeneca Pharmaceuticals Co., Ltd., National Drug approval number: J20150044), dapagliflozin was given as group B, and metoprolol succinate sustained-release tablets were given orally, 11.875-47.5 mg/time, once a day. All three groups were treated continuously for 3 months.

### 2.5. Observation Indicators

These are as follows: (1) comparison of the levels of cardiac function ultrasound indexes. Left ventricular end diastolic diameter (EDD), left ventricular ejection fraction (LVEF), and end systolic diameter (ESD) were estimated by Siemens PRIME ACUSON ES2000 and Philips EPIQ 7C Doppler ultrasound. (2) Comparison of myocardial infarction area. Myocardial ECT was used to reconstruct the tomographic images of the heart in three mutually vertical directions: horizontal long axis, vertical long axis, and short axis. The infarction area components of each tomography were measured and recorded as *S*_*x*_, *S*_*y*_, and *S*_*z*_, and the total infarct area was recorded as *S*. According to $S=\sqrt{\left(S_{x}^{2}+S_{y}^{2}+S_{z}^{2}/2\right)}$, *S*_*x*_ is the infarct area component in the long axis direction, *S*_*y*_ is the infarct area component in the short axis direction, and *S*_*z*_ is the infarct area component in the horizontal axis direction. The calculation method of *S*_*x*_ was to measure the length of the damaged myocardium on the long axis of each tomographic image, respectively, as *A*_1_*B*_1_, *A*_2_*B*_2_, *A*_3_*B*_3_ ⋯ *A*_*n*_*B*_*n*_, and the vertical distance between adjacent tomographic image was denoted as *d*, *S*_*x*_ = (*A*_1_*B*_1_ + *A*_2_*B*_2_) × *d*/2 + (*A*_2_*B*_2_ + *A*_3_*B*_3_) × *d*/2 + ⋯⋯. The algorithm of *S*_*y*_ and *S*_*z*_ was the same as that of *S*_*x*_, and the myocardial infarction area was compared between the three groups at 3 months postoperation. (3) Comparison of the levels of inflammatory and oxidative stress indexes in all three groups. Venous blood (5 ml) was collected from each patient in fasting before and after treatment and then centrifuged at 2500 r/min for 15 min, and then, the supernatant was removed and cryopreserved for testing. The serum levels of interleukin-6 (IL-6) and high-sensitivity C-reactive protein (hs-CRP) were determined by the Enzyme-Linked Immunosorbent Assay (ELIZA). The serum levels of malondialdehyde (MDA) and superoxide dismutase (SOD) were determined by double-antibody sandwich ELIZA. (4) Comparison of the serum levels of N-terminal probrain natriuretic peptide (NT-pro BNP), lipoprotein (a) (Lp(a)), ischemia-modified albumin (IMA), and secreted frizzled-related protein 5 (SFRP5) in all three groups. The serum levels of NT-pro BNP, IMA, and SFRP5 were determined by ELIZA, and the Lp(a) level was measured by automatic biochemical analyzer. (5) Comparison of the onset of adverse effects among all groups. (6) Comparison of the occurrence of cardiovascular adverse events among the three groups.

### 2.6. Statistical Methods

To process and analyze the data, statistical software (SPSS 20.0) was used. Data of measurement were represented as *x̅*±*s*. For intergroup comparison, an independent sample *T*-test was applied. To compare before and after treatment effects, paired *T*-test was applied. *χ*^2^ test was used for comparison. Count data represented as frequency and constituent ratio. *P* < 0.05 was considered statistically significant.

## 3. Results

### 3.1. Comparison of Cardiac Function Ultrasound Index Levels among the Three Groups

No significant difference was found in LVEF, EDD, and ESD levels (*P* > 0.05) before treatment. However, the levels of LVEF and EDD in groups A and B were increased significantly after treatment, while the levels of EDD and ESD decreased. The improvement degree of LVEF and EDD levels in groups A and B was greater compared to group C (*P* < 0.05) as indicated in Table 1.

### 3.2. Comparison of Myocardial Infarction Area 3 Months after Operation among the Three Groups

There was no significant difference in the myocardial infarction area 3 months after operation among the three groups (*P* > 0.05), as shown in Table 2.

### 3.3. Comparison of Inflammation and Oxidative Stress Levels among the Three Groups before and after Treatment

Before treatment, no significant difference was found in the levels of SOD and MDA and hs-CRP and IL-6 between all groups (*P* > 0.05). The serum concentrations of MDA and hs-CRP and IL-6 were decreased after treatment in all three groups; however, the SOD level was increased. The improvement degree of serum hs-CRP, IL-6, SOD, and MDA levels in groups A and B was greater than that in group C, and the improvement degree of serum hs-CRP, SOD, and MDA was higher in group A compared to group B (*P* < 0.05), as indicated in Table 3.

### 3.4. Comparison of Serum IMA, NT-proBNP, and Lp(a) Levels among the Three Groups

Before treatment, no significant difference was found in the levels of IMA, NT-proBNP, Lp(a), and SFRP5. The levels of IMA, NT-proBNP, and Lp(a) were decreased in all groups after treatment, while the levels of SFRP5 were increased. The improvement in the serum levels of IMA, NT-proBNP, Lp(a), and SFRP5 was higher in both groups A and B compared to group C. The improvement in serum levels of IMA, NT-proBNP, Lp(a), and SFRP5 was increased in group A than in group B (*P* < 0.05) as indicated in Table 4.

### 3.5. Comparison of the Occurrence of Adverse Reactions among the Three Groups

No adverse effect was observed in all three groups.

### 3.6. Comparison of Cardiovascular Adverse Events 3 Months after Surgery among the Three Groups

The total occurrence of cardiovascular adverse reactions such as stent thrombosis, cardiac failure, ventricular fibrillation, and death was 10.71% in group A, 25.00% in group B, and 53.75% in group C. The onset of cardiovascular adverse effects 3 months postoperation was significantly different among the three groups (*χ*^2^ = 12.757, *P* < 0.05) as indicated in Table 5.

## 4. Discussion

Dapagliflozin is a novel sodium-glucose cotransporter 2 inhibitor, which was initially marketed as a hypoglycemic drug in China. However, in subsequent studies, dapagliflozin was found to have antihypertensive and diuretic effects, improve osmotic pressure, inhibit myocardial fibrosis, improve myocardial energy metabolism, and improve myocardial homeostasis in addition to hypoglycemic effects [10, 11]. In addition, dapagliflozin can reduce the body mass of patients, 60%~70% of which is adipose tissue, including visceral tissue and subcutaneous tissue, and reduce the accumulation and inflammation of epicardial adipose tissue, which can be used for the treatment of cardiovascular diseases [12]. At present, the mechanism of dapagliflozin in the treatment of cardiovascular diseases has not been fully clarified, which may include a variety of mechanisms. The initial study believed that dapagliflozin could reduce the toxicity of glucose to the heart through the hypoglycemic effect, so dapagliflozin is used more in patients with cardiovascular disease complicated by diabetes [13–15]. Studies suggest that dapagliflozin may increase the synthesis of the hepatic ketone body, enhance myocardial energy metabolism, and improve cardiac function. In addition to the common hypoglycemic effects, dapagliflozin also has the effects of hypotension, diuresis, improvement of ventricular remodeling, and myocardial cell homeostasis. Besides, it can also improve arterial stiffness, which is beneficial to the treatment of cardiovascular diseases [16]. Metoprolol sustained-release tablets are selective *β*1-receptor blockers with antisympathetic effects, which can block myocardial inflammatory response caused by receptor activation and reduce ventricular remodeling. In addition, the use of beta-blockers can reduce cardiac oxygen consumption and improve myocardial perfusion in patients with cardiovascular disease. However, the application of *β*-blockers can cause hemodynamic instability and lead to severe bronchial asthma, and the dosage of *β*-blockers is limited [17–19]. In this study, the combined application of dapagliflozin and metoprolol may reduce the dose of metoprolol sustained-release tablets and also decrease the onset of complications by ensuring therapeutic effects.

Coronary atherosclerotic plaque rupture and accompanying mural thrombus may be the main pathogenesis of acute coronary syndrome (ACS), and the activation of inflammatory response may be the main factor leading to atherosclerotic plaque instability [20]. Serum hs-CRP, IL-6, SOD, and MDA levels can indicate the degree of inflammatory response and oxidative stress response in acute myocardial infarction patients [21]. In the present study, the level of LVEF in groups A and B was increased after treatment, while the levels of EDD and ESD were decreased. The improvement degree of LVEF and EDD in groups A and B was greater compared to group C. There was no significant difference in the myocardial infarction area 3 months postoperation between all groups. Serum concentrations of MDA, hs-CRP, and IL-6 were decreased after treatment in all three groups, while the levels of SOD increased. The concentrations of SOD, MDA, and hs-CRP, IL-6 were increased in the serum of both groups A and B compared to group C. Serum concentrations of SOD, MDA, and HS-CRP were higher in group A compared to group B. It indicates that dapagliflozin combined with metoprolol sustained-release tablets can effectively improve cardiac function, inflammatory response, and oxidative stress response in myocardial infarction patients post-PCI. The combined treatment group has better effect on improving inflammation and oxidative stress response than that of doxycycline alone. The improvement effect of cardiac function, inflammation, and oxidative stress in group B with dapagliflozin alone was also better compared to group C, showing that dapagliflozin may improve the cardiac function, inflammatory response, and oxidative stress in myocardial infarction patients post-PCI, but dapagliflozin in combination with metoprolol has better efficacy. Dapagliflozin and prolonged release metoprolol tablets improve cardiac function, reduce inflammation, and reduce the response to oxidative stress. The combined treatment plays a synergistic role and has a better effect on improving cardiac function. At present, no clinical study has applied dapagliflozin combined with metoprolol in patients with myocardial infarction after PCI, and the mechanism involved in this is yet to be explored.

IMA is a marker of myocardial infarction and is closely related to the degree of myocardial ischemia. It can be produced by human serum albumin during myocardial ischemia and increases rapidly when myocardial injury occurs. When the body tissue is ischemia, blood supply and oxygen supply are reduced, cells undergo anaerobic metabolism, lactic acid accumulation, and superoxide radical (O2-) formation, which is dismutated into hydrogen peroxide (H_2_O_2_) and oxygen through superoxide dismutase, and finally, IMA can be formed in the presence of metal ions. Patients after PCI are prone to myocardial ischemic injury, and IMA is a common marker of myocardial ischemia [22, 23]. NT-proBNP is the product of BNP precursor (proBNP) after cleavage into BNP, secreted by ventricular cells, which has the role of balancing water and sodium metabolism and dilating blood vessels [24, 25]. Myocardial ischemia and hypoxia can lead to increased myocardial tension and activation of excitatory neurohumoral factors and stimulate the generation of myocardial cells, leading to the increase in the level of NT-proBNP; the higher the level of serum NT-proBNP, the greater the myocardial ischemia area [26]. According to relevant studies, serum Lp(a) can induce platelet activation by promoting the formation of arterial plaque, trigger thrombosis, and accelerate the progression of coronary atherosclerosis [27]. Studies have shown that the serum level Lp(a) increases with increased coronary lesions [28]. SFRP5 can regulate lipid metabolism and inflammatory response through Wnt signal transduction pathway, which is closely related to myocardial cell injury and cardiovascular ischemic injury [29]. In this study, the levels of IMA, NT-proBNP, and Lp(a) were decreased in all three groups after treatment, while the levels of SFRP5 were increased. The improvement degree of IMA, NT-proBNP, Lp(a), and SFRP5 was higher in both the groups A and B compared to group C. The improvement degree of IMA, NT-proBNP, Lp(a), and SFRP5 levels was higher in group A compared to group B. It shows that dapagliflozin may improve the serum level of cardiac function markers in myocardial infarction patients who undergone PCI, and dapagliflozin combined with metoprolol sustained-release tablets is more effective. This may be because dapagliflozin can improve myocardial energy metabolism, improve myocardial homeostasis, and relieve myocardial ischemia and hypoxia, and metoprolol sustained-release tablets can reduce myocardial oxygen consumption and improve myocardial perfusion in cardiovascular patients; the combined application of the two can effectively improve myocardial ischemia and hypoxia and effectively regulate the serum level of cardiac function indicators. Also, we did not observe any adverse effects in all three groups, indicating that the addition of drugs in groups A and B did not cause serious adverse reactions, indicating that the medication was safe. Comparing the onset of cardiovascular adverse effects 3 months postoperation among all groups, it showed that the occurrence of cardiovascular events was 10.71%, 25.00%, and 53.75% in groups A, B, and C, respectively. It shows that dapagliflozin in combination with metoprolol can effectively reduce the incidence of cardiovascular adverse events in myocardial infarction patients post-PCI. Previously, it has been revealed that *β*-blockers improve the prognosis in myocardial infarction patients post-PCI [30]. We suggest that the dapagliflozin and metoprolol combined use had a better effect in improving prognosis.

In conclusion, dapagliflozin in combination with metoprolol may improve cardiac function, reduce the inflammatory response and oxidative stress response, improve myocardial ischemia and hypoxia state, and improve prognosis in myocardial infarction patients post-PCI, which has clinical application value. However, this study has the following shortcomings, including the small sample size and the lack of metoprolol group. In future studies, the sample size of the study should be further expanded and the metoprolol group should be set up.

## Figures and Tables

**Table 1:** Comparison of cardiac function ultrasound index levels among three groups (*x̅*±*s*).

Group	LVEF (%)		EDD (mm)		ESD (mm)	
	Before treatment	After treatment	Before treatment	After treatment	Before treatment	After treatment
Group A (*n* = 28)	46.40 ± 5.44	58.60 ± 4.47^ac^	58.86 ± 4.46	54.01 ± 4.93^ac^	47.49 ± 2.95	44.15 ± 3.31^a^
Group B (*n* = 28)	46.44 ± 5.14	57.48 ± 5.58^ac^	59.46 ± 5.14	55.22 ± 4.98^ac^	47.59 ± 4.28	45.25 ± 5.45^a^
Group C (*n* = 28)	45.10 ± 3.90	51.06 ± 4.52^a^	58.64 ± 7.80	58.13 ± 7.13	46.53 ± 4.22	46.28 ± 4.31

^a^Same group comparison before treatment (*P* < 0.05). ^b^Comparison with group B (*P* < 0.05). ^c^Comparison with group C (*P* < 0.05).

**Table 2:** Comparison of myocardial infarction area 3 months after operation among the three groups (*x̅*±*s*, cm^2^).

Group	Myocardial infarction area 3 months after operation
Group A (*n* = 28)	8.03 ± 1.66
Group B (*n* = 28)	8.87 ± 1.53
Group C (*n* = 28)	8.24 ± 2.14

^a^Same group comparison before treatment (*P* < 0.05). ^b^Comparison with group B (*P* < 0.05). ^c^Comparison with group C (*P* < 0.05).

**Table 3:** Changes in the inflammation and oxidative stress levels before and after treatment in the three groups (*x̅*±*s*).

Group	hs-CRP (mg/l)		IL-6 (ng/l)		SOD (U/ml)		MDA (nmol/l)	
	Before treatment	After treatment	Before treatment	After treatment	Before treatment	After treatment	Before treatment	After treatment
Group A (*n* = 28)	13.82 ± 2.54	6.18 ± 1.16^abc^	14.81 ± 3.29	5.84 ± 0.73^ac^	41.16 ± 4.50	64.42 ± 5.52^abc^	8.17 ± 1.85	3.37 ± 1.65^abc^
Group B (*n* = 28)	13.07 ± 2.57	7.88 ± 1.24^ac^	14.64 ± 3.71	6.15 ± 1.18^ac^	40.92 ± 5.90	59.29 ± 5.06^ac^	8.03 ± 1.62	5.30 ± 1.40^ac^
Group C (*n* = 28)	13.85 ± 3.58	10.14 ± 2.73^a^	15.12 ± 4.53	9.04 ± 1.68^a^	40.74 ± 4.13	50.33 ± 7.01^a^	8.76 ± 1.86	6.42 ± 1.58^a^

^a^Same group comparison before treatment (*P* < 0.05). ^b^Comparison with group B (*P* < 0.05). ^c^Comparison with group C (*P* < 0.05).

**Table 4:** Comparison of serum of IMA, NT-proBNP, Lp(a), and SFRP5 levels among the three groups (*x̅*±*s*).

Group	IMA (U/ml)		NT-proBNP (pg/ml)		Lp(a) (mg/l)		SFRP5 (ng/ml)	
	Before treatment	After treatment	Before treatment	After treatment	Before treatment	After treatment	Before treatment	After treatment
Group A (*n* = 28)	91.01 ± 8.68	35.64 ± 2.92^abc^	3686.42 ± 499.58	2079.91 ± 322.45^abc^	332.47 ± 37.33	264.46 ± 32.41^abc^	21.13 ± 3.72	84.03 ± 8.20^abc^
Group B (*n* = 28)	90.49 ± 7.90	42.69 ± 7.62^ac^	3670.94 ± 517.82	2411.84 ± 523.83^ac^	334.76 ± 46.72	284.89 ± 36.59^ac^	21.81 ± 2.45	59.90 ± 6.95^ac^
Group C (*n* = 28)	91.22 ± 10.03	58.62 ± 5.03^a^	3634.97 ± 451.28	2846.79 ± 415.30^a^	332.61 ± 29.12	304.22 ± 29.83^a^	22.37 ± 2.88	41.73 ± 6.19^a^

^a^Same group comparison before treatment (*P* < 0.05). ^b^Comparison with group B (*P* < 0.05). ^c^Comparison with group C (*P* < 0.05).

**Table 5:** Comparison of cardiovascular adverse events 3 months after surgery among the three groups (*n*(%)).

Group	Heart failure	Ventricular fibrillation	Death	Total incidence of cardiovascular adverse events
Group A (*n* = 28)	3 (10.71)	0 (0.00)	0 (0.00)	3 (10.71)^c^
Group B (*n* = 28)	4 (14.29)	2 (7.14)	1 (3.57)	7 (25.00)^c^
Group C (*n* = 28)	9 (32.14)	3 (10.71)	3 (10.71)	15 (53.57)

^a^Same group comparison before treatment (*P* < 0.05). ^b^Comparison with group B (*P* < 0.05). ^c^Comparison with group C (*P* < 0.05).

## Data Availability

The labeled dataset used to support the findings of this study are available from the corresponding author upon request.
